# Promoting Sustainable Green Growth through the Use of Political Institutions: The Role of the Law

**DOI:** 10.1155/2022/9009349

**Published:** 2022-09-22

**Authors:** Caixia Zou

**Affiliations:** Shanghai University of Political Science and Law, Shanghai 201701, China

## Abstract

In the era of global development, due to the destruction of the environment by traditional production, traditional industries have been forced to open the road of green growth transformation. What kind of methods that can effectively promote sustainable green growth has become one of the current research topics that has attracted much attention. Addressing this issue is very important for the green growth sector. With the in-depth research on green growth, the research on the promotion of green growth by political institutions has gradually been carried out, and its policy advantages are of great significance to solve the problem of green growth transformation. The purpose of this paper is to examine the role of law in the promotion of sustainable green growth by political institutions. Through the analysis and research of sustainable green growth, law, and logistic regression model, it can improve the level of sustainable green growth of enterprises and solve the problem that the current level of sustainable green growth of enterprises is not high. This paper analyzes sustainable green growth, the role of law, and logistic regression models and uses relevant formulas to explain them. The experimental results show that the green growth index of group A production enterprises is higher than that of group B. Legal means have played a very important role in improving the level of sustainable green growth in the promotion of sustainable green growth by political institutions. It can meet the requirements of green growth under the current SDG concept, and its sustainability has been greatly improved.

## 1. Introduction

At present, the concept of sustainable development is deeply rooted in the hearts of the people. Many traditional enterprise production methods cannot meet the increasing requirements of green growth in terms of energy efficiency and environmental protection. Green growth requires the pursuit of economic growth and development while preventing environmental degradation, biodiversity loss, and unsustainable use of natural resources. Intervention by political institutions is a national coercive measure that can effectively solve the problems encountered in the process of promoting green growth in the SDG. Due to its policy advantages, it has been applied in various fields to successfully solve various direction guidance problems. Political institutions can take macromanagement, legislative, and administrative measures, the organization of public production and the provision of public property, financial, and other interventions. The method of law's intervention in political institutions is the most direct form of existence and has far-reaching implications for the study of how the law can play a role in promoting sustainable green growth using political institutions. The concept of green growth requires forcing changes in the traditional production methods of enterprises; so, its application is of great universal value at present. In recent years, scholars have used political institutions to solve the problem of sustainable green growth, but there are relatively few applications and researches on the role of law in this regard. Therefore, this paper is significant for the study of the role of law in promoting sustainable green growth in political institutions.

At present, with the continuous advancement of the transformation of the SDG concept, more and more scholars have conducted research on promoting sustainable green growth. Among them, in order to improve people's current sustainable living level, some scholars studied the process of G-IoT to create green and sustainable living places [1]. To study the relationship between business and the environment, Bendell explored how business owners make trade-offs related to environmentally friendly innovation [2]. In order to investigate the positive impact of green power on green product innovation performance, Chang believed that machine power and moral power have positive effects on green product innovation performance [3]. Retrofitting old cities to mitigate climate change has become a global trend. Covering a variety of strategies to improve the urban environment and make the city a more livable place, some scholars have proposed that improving the quality of life of urban residents requires sociopolitical participation, public education, and government leadership [4]. Using dynamic capability theory, Singh and El-Kassar proposed an empirically tested model for green concept research [5]. However, the methods used to promote sustainable green growth are not very efficient.

Intervention through political institutions has been shown to be direct and effective in promoting green growth. In addition, some scholars have studied the impact of government spending on the country's green economic performance under the “One Belt, One Road” initiative [6]. In order to evaluate the effect of political institutions in promoting green growth and analyze which factors drive green growth, some scholars developed a comprehensive model to study the relationship between ER, TI, and regional green growth performance (RGGP) [7]. In order to explore the influence of political relevant departments on agricultural green entrepreneurship, some scholars have studied the opportunities of agricultural entrepreneurship and the role of green entrepreneurship in achieving sustainable economic growth in Nigeria [8]. To clarify the link between political institutions and green growth, researchers have found that in addition to environmental benefits, the dissemination of technologies developed through green LIFE projects may also have important economic and social impacts [9]. These methods have promoted the progress of green growth to a certain extent, but their effect on improving the level of green growth is not direct enough.

In order to solve the mentioned low level of sustainable green growth, this paper uses a logistic regression model to analyze the role of law in promoting sustainable green growth. By simulating it, it can achieve the effect of promoting energy saving and emission reduction in the production of enterprises and improving the level of green growth. The novelty of this paper is that it uses logistic regression to analyze how political institutions, law, and logistic regression models play a role in promoting sustainable green growth through the use of political institutions: the role of law. The proposed model is described. Through experiments, it is found that the application of legal methods can effectively improve the level of green growth of enterprises.

## 2. Methods

### 2.1. Content and Organization of the Paper

With the gradual promotion of SDG thinking on a global scale, the defects and deficiencies in the production of enterprises with low sustainable green growth levels have become increasingly prominent [10, 11]. The problems of low sustainable green growth production are shown in Figure 1.

As shown in Figure 1, low sustainable green growth levels are often accompanied by uncontrolled exhaust emissions and waste water emissions, resulting in severe air pollution, water pollution, and great damage to the global environment and human living space. Therefore, it is very important to improve the level of sustainable green growth [12].

Intervention by political institutions can fully make up for the insufficiency of market supervision. From a macro and overall perspective, more appropriate action on the entire macro economy can achieve a comprehensive balance between environmental protection and economic development. The survey found that current research on the role of law in promoting sustainable green growth through the use of political institutions is incomplete. Therefore, this paper presents a study of the role of law in the use of political institutions to promote sustainable green growth [13, 14]. This paper applies a logistic regression model to the analysis of the role of law in the use of political institutions to promote sustainable green growth and proposes a new model for use in the analysis of the role of law in promoting green growth. Production enterprises controlled by legal methods through experiments and data analysis have a higher level of sustainable green growth than ordinary production enterprises. The organization of the full text is shown in Figure 2.

As shown in Figure 2, this paper is composed of five parts. The first part mainly introduces the research background of the role of law in promoting sustainable green growth through the use of political institutions to draw out the problems to be solved to illustrate the purpose and significance of this paper. Then, it makes a general analysis of the research status of the sustainable green growth field and the research field of political institutions promoting green growth and explains the content and innovation of this paper; the second part describes the organization structure and method of the whole paper, introduces the related method content of the logistic regression model, and describes the proposed logistic regression model; the third section details the data sources used for the study Promoting Sustainable Green Growth through the Use of Political Institutions: the Role of the Law; the fourth part is experimental analysis through the experimental analysis of the production consumption and energy consumption of different groups of enterprises, the production emissions of different groups of enterprises, and the level of sustainable green growth of different groups and draws conclusions after analyzing the result data; the fifth part is the conclusion.

### 2.2. Logistic Regression Model

In this paper, logistic regression is chosen for the analysis of relevant data in the study of the role of law in promoting green growth through the use of political institutions. Logistic regression is a special kind of linear model, which is a special form of the normalized linear model [15, 16]. Both logistic regression and linear regression are generalized linear models. Specifically, linear models derived from the exponential family of distributions. Linear regression is based on the premise that *Y*|*X* follows a Gaussian distribution. Logistic regression is based on the premise that *Y*|*X* follows the Bernue distribution. As shown in Figure 3, applying the logistic regression model to the relevant data analysis on the role of law in promoting green growth can yield better results [17].

Its advantages are that it is very simple to implement first, and secondly, it has a wide range of applications, less classification and calculation, fast speed, and easy understanding. In contrast to linear regression, logistic regression uses a logistic function to map the range of dependent variables from the actual range 0 to 1. Logistic regression is basically used for classification problems [18]. The former can only be used for regression problems, while the latter is used for classification problems (2-class, multiclass). Linear regression has no link function or does not work. The link function of logistic regression is a logarithmic probability function; linear regression uses the minimum square method as the parameter estimation method, and logistic regression uses the most-likelihood method as the parameter estimation method.

When a relevant dataset {M_*i*_,_*i*_|*l*_*i*_ ∈ {0, 1}, *i* = 1, . ⋯ , *z*} is available on the role of law in promoting sustainable green growth through political institutions, there is formula (1):

(1) $$\begin{array}{c} M\vartheta =\overset{z}{\underset{i=1}{\sum }}l_{i}^{Y}\vartheta . \end{array}$$

Among them, *l*_*i*_ ∈ *T*^*e*^, *ϑ* ∈ *T*^*e*^.

To get the logistic regression model of the relevant data, a hypothesis function must firstly be constructed as shown in formula (2):

(2) $$\begin{array}{c} {\text{N}}_{\vartheta }\left(l\right)=\text{G}\left(l^{Y}\vartheta \right)=\frac{1}{1+\exp{\left(-l^{Y}\vartheta \right)}^{\prime }}. \end{array}$$

N_*ϑ*_(*l*) is the constructed hypothetical function that affects the green growth level; G(*x*) = 1/1 + exp(−*x*) is the logistic function.

Both function *J*_*δ*_(*a*) and logic function *h*(*x*) are assumed to have values between 0 and 1.

In the green growth related data set {M_*i*_,_*i*_|*l*_*i*_ ∈ {0, 1}, *i* = 1, . ⋯ , *z*}, the influence on the green growth level is set as the dependent variable, and the conditional probability when its value is 1 can be expressed by formula (3):

(3) $$\begin{array}{c} \text{Y}\left(b=1\left|l,\vartheta \right.\right)=N_{\vartheta }\left(a\right)=\frac{1}{1+\exp\left(-l_{i}^{Y}\vartheta \right)}=y. \end{array}$$

Conversely, the conditional probability when the dependent variable is 0 can be expressed by formula (4):

(4) $$\begin{array}{c} \text{Y}\left(b=0\left|l,\vartheta \right.\right)=1-N_{\vartheta }\left(l\right)=1-y. \end{array}$$

According to the discussion, both sample data M ∈ *T*^*z*×*y*^ and class label *G* ∈ *T*^*z*^(*b*_*i*_ ∈ {0, 1} conform to Bernoulli distribution.

By integrating these formulas, the logistic regression model affecting the level of green growth can be obtained as shown in formula (5):

(5) $$\begin{array}{c} \text{R}\left(b\left|l,\vartheta \right.\right)=y^{b}{\left(1-y\right)}^{\left(1-b\right)}. \end{array}$$

C(*b*|*x*, *ϑ*) is the probability that the sample l belongs to the condition of class b; *ϑ* is the parameter vector of the variable.

The company's sustainable green growth level evaluation index is set as a nominal variable, and the company is investigated in the form of whether the intervention items implemented by the company affect the company's sustainable green growth level. Therefore, the logistic regression model is used to analyze the factors affecting the evaluation index of sustainable green growth level [19]. Assuming that the probability of occurrence of an impact on the sustainable green growth level of the enterprise is *C*, and the value range is 0 to 1, the probability that the event does not occur is 1 − *C*. This probability can be calculated using a logistic regression function [16]. The expression is formula (6):

(6) $$\begin{array}{c} Ln\left(\frac{C_{1}}{1-C_{1}}\right)=\psi_{0}+\psi_{1}b_{1}+\psi_{2}b_{2}+\cdots +\psi_{i}b_{i}\left(i=1,2,3,\cdots ,n\right). \end{array}$$

*C*_1_ is the probability of a positive impact, *ψ* is a constant term, *ψ*_*i*_ is the regression coefficient of the *i*-th factor affecting sustainable green growth, and *b*_*i*_ is the *i*-th independent variable.

According to the problems of today's low sustainable green growth level, presuppositions are made for the factors affecting an enterprise's sustainable green growth level. It is assumed that the energy consumption of the enterprise, waste emissions, output indicators, and production methods can be affected by legal control. Through the aspects of formulation of relevant tax policies in legal methods, formulation of relevant emission guidelines, energy use regulations, and so on, the deterministic factors for improving the level of green growth can be obtained through data investigation and analysis of these factors. At the same time, it determines the role of law in promoting sustainable green growth and adjusts the production-related items of enterprises through legal methods to better guide production enterprises to improve the level of sustainable green growth. After assigning the preset attributes into the initial model, a complete and sustainable green growth level factor influencing model can be obtained. The influence coefficient of each item is obtained, and the conclusion is drawn after analysis in Experimental Analysis.

## 3. Experimental Analysis

There are two main parts of the data used for the analysis of this experiment. On the one hand, it collects data on the experimental data on the use of political institutions to promote sustainable green growth: the role of law among middle and senior managers in 10 selected production enterprises in the form of a questionnaire survey. Among them, 300 questionnaires were issued, 286 questionnaires were recovered, 284 were valid questionnaires, and the recovery rate was 94.6%. The collected information data are mainly the basic information characteristics of the enterprise: the production situation of the enterprise. Examples of the specific content of the collected information are shown in Tables 1 and 2.

The object of this part of the dataset consists of three attributes, namely, the age of the manufacturer, the type of property rights of the manufacturer, and the type of production of the manufacturer.

The subitems included in this part are annual gross output value (unit: million yuan), annual standard energy consumption (unit: million tons), annual carbon emissions (unit: million tons), and annual carbon emission intensity (it is the carbon emission per million output value, and the unit is ton/million yuan).

At the same time, an expert group is established to evaluate the level of green growth by analyzing and discussing the collected corporate data. Examples of the evaluation criteria are shown in Table 3.

Among them, in view of the energy loss, energy utilization efficiency, the “three wastes” in the discharge process, the degree of environmental pollution, and the output efficiency of the production enterprises, the scoring rules are formulated and adopted after testing. The expert group scored the production enterprise's energy consumption, environmental protection, sustainability, and output, with a total of 10 points. The higher the score, the higher the green growth level of the item.

After a 6-month test in this experiment, several enterprises were divided into observation group A, which were production enterprises that were intervened and controlled through legal methods. The legal method adopted was to restrict the use of its resources, restrict its emissions, and make new plans for its production targets through the formulation of legal regulations; enterprises of group B were ordinary production enterprises without control. The following conclusions are drawn from the collected information related to the production situation of the enterprise, the environmental pollution situation, and the level of sustainable green growth.

### 3.1. Production Consumption and Energy Consumption of Different Groups of Enterprises

The collected information on production and energy consumption of the enterprise is compared among different groups, and the specific content of the result analysis is shown in Figure 4.

As can be seen from Figure 4, overall, the energy consumption of group B enterprises is higher than that of group A enterprises. The annual consumption of coal washing by group B enterprises has reached 2.7614 million tons, which is twice as high as that of group A enterprises. The production consumption of this enterprise is very large. Judging from the overall consumption growth of different groups of production enterprises during the test period, with the increase of time, the energy consumption rate of group A slowed down significantly, and the total consumption was lower than that of group B, with a difference of nearly 23.44%. This is due to the adjustment of the energy use of group A enterprises through legal control to make it optimize the energy use method and improve the energy utilization rate. Legal control can help enterprises save energy consumption in production.

### 3.2. Production Emissions of Different Groups of Enterprises

The collected data on the production and emission of different groups of enterprises are compared and analyzed, and the specific content of the results is shown in Figure 5.

Figure 5 The emissions of “three wastes” of group A enterprises are significantly lower than those of B renting enterprises. During the experiment, the total production emissions of group A enterprises initially increase faster than that of group B enterprises, reaching 2,765,800 tons, and then begin to decline again in the next two months, reaching only 1,371,500 tons. Group companies are less than half. This is because, under the constraints of laws and policies, the enterprises in group A firstly improve production efficiency through technological innovation, concentrate production emissions in the early stage to achieve production tasks, and gradually reduce production emissions in the later stage. Intervening in the production emissions of enterprises through legal methods can effectively reduce production emissions.

### 3.3. Different Sets of Sustainable Green Growth Levels

After analyzing and processing the data of each enterprise through the data analysis model, the expert group conducts an overall assessment of the sustainable green growth level of different groups of enterprises, and the specific results are shown in Figure 6.

Figure 6 On the whole, the sustainable green growth level of group A is significantly higher than that of group B. Among various evaluation indicators, although the score of group B enterprises in productivity is 8.31, it is higher than that of group A enterprises. However, the scores in the other three evaluation indicators are lower than those of group B enterprises. Therefore, in the comprehensive evaluation, the companies in group A achieved 8.69 points, and the companies in group B only scored 6.83 points. After controlling the green growth-related indicators produced by company A through legal methods, the sustainable green growth level of this group of companies has been improved.

## 4. Conclusion

Sustainable green growth under SDG is becoming more and more intense, and people's requirements for green growth are getting higher and higher. The development of sustainable green growth is inseparable from the contributions of political institutions and laws. Laws have been widely used in many fields because of their direct intervention advantages. Through comprehensive experimental analysis, group A companies that use legal methods to manage and control are better than group B companies that do not use political agency intervention in various indicators of sustainable green growth. They are not only more sustainable but also better. The production of legally controlled enterprises is used to meet the needs of sustainable green growth. There may be some uncertain factors, such as the instability of the use environment and the difference of operators, so that the results of this experiment are not completely accurate and reliable, and there are certain differences. This paper firstly analyzed the use of political institutions to promote sustainable green growth, laws, and logistic regression and then analyzed their function using related principal formulas. Then, in the experimental part, this paper compared the production enterprises that use legal intervention and those that do not use legal intervention. The conclusion is that the sustainable green growth level index of the production of enterprises that are controlled by legal methods is higher than that of ordinary production enterprises, and the sustainability is more stable. Therefore, a study of promoting sustainable green growth using political institutions is as follows: the role of law is necessary.

## Figures and Tables

**Figure 1:** Problems with low sustainable green growth production.

**Figure 2:** Full-text content organization.

**Figure 3:** Data analysis based on logistic regression model.

**Figure 4:** Production consumption and energy consumption analysis of different groups of enterprises.

**Figure 5:** Analysis of production emissions of different groups of enterprises.

**Figure 6:** Evaluation of the sustainable green growth level of different groups of enterprises.

**Table 1:** Examples of basic characteristic information content of some manufacturers in the questionnaire survey.

Project	Enterprise 1	Enterprise 2	Enterprise 3
Business age	7	6	11
Property rights	Privately held	Collective holding	Foreign trade holding
Production type	Extractive	Assembly type	Decomposition type

**Table 2:** Examples of production information content of some manufacturers in the questionnaire survey.

Project	Enterprise 1	Enterprise 2	Enterprise 3
Annual output value	7.64 million	3.40 million	11.41 million
Annual energy consumption	34.15million tons	18.64 million tons	117.28 million tons
Annual carbon emissions	13.14 million tons	5.27 million tons	26.96 million tons
Annual carbon intensity	11.24	9.61	23.15

**Table 3:** Examples of the content of the evaluation of the green growth level of some enterprises by the expert group.

Index	Enterprise 1	Enterprise 2	Enterprise 3
Energy saving	3.64	7.54	4.51
Environmentally friendly	4.51	6.35	2.45
Sustainability	4.91	6.14	3.77
Productivity	7.64	5.46	8.63
Comprehensive index evaluation	5.14	7.38	4.76

## Data Availability

The data used to support the findings of this study are available from the corresponding author upon request.
